# The Efficacy of Combined Therapy of Regorafenib with Detoxicating and Stasis Softening Chinese Herbal Spleen Tonics in Mid-/Late-Stage Hepatocellular Carcinoma

**DOI:** 10.1155/2022/9316873

**Published:** 2022-06-06

**Authors:** Yaokai Ma, Guowei Liu, Jinzu Yang, Xin Li, Xiyi Yang, Shiming Fang, Baocheng Zhao

**Affiliations:** ^1^Intervention Department, Shanghai Xuhui Central Hospital, Shanghai, China; ^2^Department of Oncology, Shanghai Longhua Hospital, Shanghai, China

## Abstract

**Objective:**

To explore the efficacy of combined therapy of Regorafenib with detoxicating and stasis softening Chinese herbal spleen tonics (DSS-splenic tonics) in mid-/late-stage hepatocellular carcinoma.

**Methods:**

Retrospective observational data of 120 patients were obtained, 60 of which received combined therapy of DSS-splenic tonics and regorafenib. Adverse event, overall survival (OS), and time-to-progress (TTP) were analyzed. Synergistic effect of DSS-spleen tonics was found and validated in human hepatocellular carcinoma HCCLM3 cell line and xenograft mouse models.

**Results:**

Combination of regorafenib and DSS-splenic tonics also slightly extended the TTP and OS compared with treatment of regorafenib alone, suggesting DSS-splenic tonics has synergistic effect with regorafenib. Both Regorafenib and DSS-spleen tonics exerted inhibitory effect on cell viability and invasion capability of HCCLM3 cells, and combining both could enhance the antitumor effect. At molecular level, we found that VEGF, HIF-1*α*, MVD, and VEGF2 were all suppressed by regorafenib and DSS-splenic tonics. These results suggest that DSS-spleen tonics function synergistically with regorafenib in HCC by enhancing the regulation of regorafenib on VEGF, MMP-2, HIF-1*α*, and MVD, and may diminish angiogenesis during HCC progression.

**Conclusion:**

DSS-spleen tonics could exert synergistic antitumor effect with regorafenib via targeting VEGF.

## 1. Introduction

Hepatocellular carcinoma (HCC) is a common malignancy ranking in top five with regards to mortality [1, 2]. China is the most inflicted country by HCC accounting for 55% incidence and 45% death all over the world, and HCC becomes the topmost killer for those younger than 60 years of age [3, 4]. HCC patients in China are often complicated with other hepatic illness such as hepatitis and cirrhosis, or even presenting slow lipiodol deposition and high tumor heterogeneity, which undermines the efficacy of TACE [5, 6]. However, the access to new technologies, such as Radio-Frequency Ablation (RFA), Microwave Ablation (MWA), cryoablation, and radiotherapy, is limited to certain indications, hindering the extensive application of these approaches [7, 8].

Chemotherapy and target therapy are two of the few effective systemic therapies of cancer, while liver cancer cells are often insensitive to chemotherapeutic drugs which usually bring about severe side effects, further decreasing the patient adherence [9, 10]. Sorafenib demonstrated not only relatively low objective remission rate (ORR) but also severe adverse events, which yielded very limited clinical benefits [11, 12]. However, its affordability and the lack of clinical trial in Chinese population limit its accessibility. Therefore, mid/late-stage HCC patients moderately benefit from modern medical therapies.

The approach of Chinese traditional medicine has unique characteristics different than the modern medicine, which addresses the disease from holistic aspect and usually focuses on improving the functionality of loci affected by the diseases [13]. There has been therapeutic paradigm in Chinese traditional medicine hospital that integrates modern medicine and Chinese traditional medicine, treating the cancer while nourishing and rejuvenating the organs or tissues hampered by the disease or the treatment [14, 15]. Chinese traditional medicine proposed that spleen is an organ that should be nourished when treating the cancer, which has achieved desirable efficacy in combining both traditional medicine with modern medicine to treat HCC [16]. We formulate a prescription by mixing the water extracts of a series of Chinese traditional herbal medicines, which was intended to nourish the spleen during cancer treatment and thus was called detoxicating and stasis softening Chinese herbal spleen tonics (DSS-spleen tonics). This study conducted a retrospective assessment of the efficacy of combined therapy of DSS-spleen tonics with target therapy in a multicenter cohort study and validated the underlying effector in cell line and primary HCC xenograft mouse models. The improved efficacy was observed in HCC xenograft models administrated with Regorafenib and DSS-spleen tonics combined than single therapy of Regorafenib. Our study provides both evidence-based and mechanism for combined therapy of tyrosine kinase inhibitor drugs in HCC.

## 2. Material and Methods

### 2.1. Plan

#### 2.1.1. Formula of DSS-Spleen Tonics

The DSS-spleen tonics comprise of extracts of the following herbals: *Radix pseudostellariae*, Radix Pearl Ginseng, fried Atractylodes rhizome, Poria, orange peel, chicken gizzard lining, hawthorn, Tianlong, Zedoary Curcuma, peach kernel, Thunberg Fritillary Bulb, cypress on stone, hibiscus leaf, *Radix astragali*, Angelica.

#### 2.1.2. Patients and Treatment

The patients with advanced HCC recurred after first-line treatment of sorafenib at eight Chinese hospitals from August 2016 to August 2018 were selected for this study. Their medical records were retrieved from the hospital's Health Information System. This study was initiated in May 2019. As per the label of regorafenib treatment, only the patients with normal renal and liver function and bone marrow. The disease progression were confirmed by experienced radiologist, and the sorafenib tolerability was confirmed. The treatment cycle is composed of 3 weeks of oral administration of regorafenib at starting dose 160 mg, QD (once a day), and 1 week of no treatment. Reduced starting dose may apply for some patients depending on their clinical manifestation and adverse events, and the recommendations for metastatic colorectal cancer and gastrointestinal cancer was adopted. A subset of patients received 300 ml DSS-spleen tonics 5 hours after regorafenib administration, once a day for 4 days. Alpha-fetoprotein (AFP), radiological assessment, Child-Pugh class, Barcelona Clinic Liver Cancer (BCLC), Eastern Cooperative Oncology Group performance status [ECOG-PS] were collected for each patient.

All procedures performed in studies involving human participants were in accordance with the ethical standards of the Ethnic Committee of the Shanghai Xuhui District Central Hospital. As this is a retrospective study, thus local ethic committee approval was not required. All the patients gave their written information consent.

#### 2.1.3. HCCLM3 Cell Culture

The HCCLM3 cell line was procured from Institute of Liver Cancer Research of Fudan University Affiliated Zhongshan Hospital. High glucose Dulbecco's modified Eagle's media (DMEM, Thermofisher Scientific, Waltham, USA) supplemented with 10% fetal bovine serum (Thermofisher Scientific, Waltham, USA) was used to culture the cells. The incubator was maintained at 37°C, 5% CO_2_.

### 2.2. Data and Index

#### 2.2.1. MTT Assay

The cell viability was measured with MTT assay; 7 × 10^3^ HCCLM3 cells were seeded in each well of 96-well plate (BD Falcon, Franklin Lakes, NJ). Cells were allowed to be attached to the well wall overnight at 37°C 5% CO^2^. A measure of 10 *μ*l MTT in phenol red-deficient DMEM was added to each well, and the plates were incubated at 37°C for 3 hours. The active enzymes of viable cells catalyzed the yellow MTT into purple formazan crystals during the incubation. After removal of the top medium, the formazan crystals were dissolved in isopropanol. Absorbance at 570 nm was measured by SpectraMax fluorescence multiwell plate reader (Molecular Devices, Sunnyvale, CA).

#### 2.2.2. Western Blot

Radioimmunoprecipitation assay buffer (RIPA) was used to extract proteins from cells, which were separated by 10% sodium dodecylsulfate-polyaclylamidegel electrophoresis (SDS-PAGE) and then transferred to polyvinylidene fluoride (PVDF) membranes. The membranes were blocked with 5% skimmed milk resolved in PBS (pH 7.4, with 0.1% Tween 20) for 60 min. Afterward, primary antibodies was added to the membrane which were incubated at 37°C for 60 minutes. After removal of excess primary antibody, horseradish peroxidase (HRP)-linked secondary antibody diluted in 0.01 M PBS was added to the membrane and incubated at room temperature for 30 min, and then washed with 0.01 M PBS for four times. Enhanced BM chemiluminescence blotting substrate (Roche Diagnostics) was used to detect the antigens. The luminescence intensity was quantified by Image J. mouse-anti-human HIF-1*α* (1:250, Sigma-Aldrich), MMP-2 (1:1000, Sigma-Aldrich), VEGF (1:1000, Sigma-Aldrich), and MVD (1:1000, Sigma-Aldrich).

## 3. Results

### 3.1. Clinical Characteristics of Recruited Patients

Retrospective clinical data of 120 patients were collected from the database of Shanghai Longhua Hospital. The age of recruited patients fell between 28 and 70, and median is 48 years of age. There are 92 male patients and 28 female patients, and 70% of them were type hepatitis B, 10% were hepatitis C, and the remaining were undetermined hepatitis. BCLC staging differentiate 15% as B (mid) stage and 85% as C (late) stage. Around 62% patients manifested with vascular invasion, and 30% presented extrahepatic metastasis. Those 120 patients were stratified based on baseline characteristics and allocated into three study groups randomly, ensuring each clinical characteristic were evenly distributed within the same group. There were 40 patients receiving single treatment of regorafenib (REG) as second-line treatment and the other 40 received combined therapies of regorafenib and DSS-spleen tonics (REG-DSS). BCLC staging, ECOG performance status, Child-Pugh class, histological, and radiological assessments were used to characterize tumor status. Tumor biomarker AFP, AFP-L3, *α*-L fucosidase, and abnormal prothrombin were collected to assist the definition of tumor progression or recession. Survival time and follow up were documented to analyze the survival rate. Overall survival was used to measure the efficacy, which was defined as the date of diagnosis as B/C stage HCC and the end date of follow up or death. Baseline characteristics were summarized in Table 1, and the adverse events during the treatment cycles were recorded in Table 2.

Most patients had Child-Pugh class A cirrhosis, and 63% of the patients were classified as BCLC staged B, and rest of them were stage C at baseline. Diarrhea, fatigue, palmar-plantar erythrodysesthesia, elevated aspartate aminotransferase, decreased appetite, and hypertension were the most common adverse events (AE) (Table 2). In REG group, 32 patients required dose modifications, with manifestation of palmar-plantar erythrodysesthesia, decreased appetite, fatigue, and elevated AST (*Aspartate aminotransferase*). In REG-DSS group, 34 patients had reduced dose of both REG and DSS, the most common clinical manifestation for dose modification are fatigue, decreased appetite, palmar-plantar erythrodysesthesia, and elevated AST.

During treatment cycles, both groups did not show significant difference in occurrence of AE, nor did they present difference in the distribution of AEs, indicating that DSS may not alter the safety profile of regorafenib (Table 2). Note worthily, the incidence of palmar-plantar erythrodysesthesia is slightly reduced in DSS group, implying protective effect of DSS.

Overall, the median Time to Progression (TTP; time from randomization to objective tumor progression), progression-free survival (PFS; time from randomization to first occurrence of disease progression or death from any cause) and overall survival in the totally 120 patients were 7.1 months (95% CI 3.5–9.8), 7.1 months (95% CI 3.5–9.8), and 17.6 months (95% CI 11.5–22.8), respectively. We next sought to examine how the treatment duration would impact the efficacy. Each treatment group was further divided into two groups based on treatment duration, respectively. The cutoff treatment duration was 4.2 months. The patients with treatment duration longer than 4.2 months had significantly longer TTP and PFS than those with treatment duration below 4.2 months, 7.6 months (95% CI 6.6–8.5) vs. 4.3 months (95% CI 2.0–6.5) (Table 3). Within REG group, patients with treatment duration longer than 4.2 months had significantly longer TTP and PFS than those with treatment duration below 4.2 months, 7.1 (95% CI 5.8–8.6) vs. 3.7 months (95% CI 2.5–4.8); Within REG-DSS group, patients with treatment duration longer than 4.2 months had significantly longer TTP and PFS than those with treatment duration below 4.2 months, 7.9 (95% CI 6.8–8.9) vs. 4.6 months (95% CI 3.2–6.2). Compared with REG group, REG-DSS group has slightly longer TTP (6.8 vs. 7.3, Table 3), indicating that DSS might potentiate the antitumor effect of regorafenib. During the observation period, 18 patients died and the median overall survival (OS; time from randomization to death from any cause) for the total 120 patients were 18.8 (95% CI 12.6–20.5) months. DSS group demonstrated slightly longer median OS than REG group, suggesting DSS may enhance the efficacy of regorafenib (Table 3).

Given the retrospective results of above observation, we next sought to examine the effect of DSS-spleen tonics in human hepatocellular carcinoma cell line. HCCLM3 was employed for cellular study by the courtesy of Institute of Cancer Research, Fudan University Affiliated Zhongshan Hospital. HCCLM3 cell lines were cultured in regorafenib and/or DSS-spleen tonics. Cell proliferation was evaluated by MTT assay at 24, 48, and 72 hours posttreatment. As shown in Figure 1(a), the overall cell count began to differentiate after 24 hours, where combined use of DSS and regorafenib showed inhibited cell growth than regorafenib alone. All treatments have slower cell proliferation than control. In Transwell assay, the inhibitory effect of regorafenib presents correlation with the administrated concentration, and control has the most infiltrated cells (Figure 1(b)). Similarly, cotreatment of DSS-spleen tonics showed enhanced antitumor effect on cell invasion (Figure 1(b)).

DSS-spleen tonics had synergistic antitumor efficacy with regorafenib in human HCCLM3 xenograft nude mice model.

We established an HCC model by injecting HCCLM3 cells into healthy male athymic BALB/c (nu/nu) nude mice and transplanting the developed tumor into the liver of a new nude mice. A total of 40 xenograft nude mice model were evenly randomized into four groups and treated with the following drugs: DSS-spleen tonics (group A), regorafenib (group B), DSS-spleen tonics + Reorafenib (group C), and saline control (group D). The weight of mice and the size of subcutaneous tumor were measured daily to assess the efficacy of treatments. Before treatment, the mean body weight of group A, group B, group C and control were 17.8 ± 0.79 g, 17.9 ± 0.88 g, 17.8 ± 0.79 g, and 18.7 ± 0.74 g. After treatment, the mean body weight of group A, group B, group C, and control were 21.94 ± 1.11 g, 21.63 ± 1.00 g, 25.67 ± 0.87 g and 20.64 ± 1.07 g (Tables 4 and 5). The body weight increase of group C is more significant than group A and group B (Figure 2(a)).

Mice in the experimental groups presented better mental status than the control. One week posttreatment, each group has a mouse displaying subcutaneous metastatic mass, in which the group C mouse undergone decreasing size of metastatic mass and the mass disappeared. The other groups undergone decreasing size of tumor as well, and the tumor size were eventually maintained at a small level but never disappeared (Figure 2(b)). As shown in Table 4, the tumor weight of groups A, B, C, and D (control) were 2.66 ± 0.32 g, 2.54 ± 0.41 g, 0.95 ± 0.61 g, and 3.69 ± 0.34 g. Lung tissue were obtained to evaluate the lung metastasis of HCC mice model. We found that group C demonstrated markedly less mass in the lung (Figure 2(c)).

Lung tissues were obtained from the mice model. Histological assay showed that all experimental groups did not have metastasis compared to lung metastasis in control group (Figure 2(d)). Taken together, these results suggest that combined use of DSS-spleen tonics and regorafenib could significantly improve the efficacy of regorafenib.

After cell line and *in vivo* validation of the antitumor effect of DSS-spleen tonics, we next investigate the underlying molecular mechanism. We performed immunochemistry histology assay of the tumors obtained from xenograft. Interestingly, the vascular endothelial growth factor (VEGF), HIF-1*α* (Hypoxia Inducible Factor-1), microvascular decompression (MVD), and vascular endothelial growth factor-2 (VEGF-2) were all underexpressed in group A, B, and C, compared with control suggesting that DSS-spleen tonics and Regorafenib share the same target in HCC xenograft model (Figure 3(a)). RT-qPCR and Western blot were then used to validate the regulation of DSS-spleen tonics on expression of VEGF, HIF-1*α*, VEGF2, and MVD. As shown in Figure 3(b), the expression of these molecules were significantly reduced in the experimental groups, and combined use of DSS-spleen tonics and Regorafenib demonstrated the most significant decrease at both transcriptional and translational levels, suggesting that DSS-spleen tonics has synergistic anti-tumor effect with Regorafenib.

## 4. Discussion

Liver cancer ranks fourth in the most common causes of cancer-related death and have high incidence worldwide. World Health Organization estimates the mortality due to liver cancer will reached 1 million in 2030 as per the current annual projections [17]. Hepatocellular carcinoma (HCC) is a major type of liver cancer that originates from hepatitis B or C virus (HBV or HCV) infection, alcohol abuse, or even NAFLD [18]. Mid/late stage HCC are not subject to or recur from resection, ablation or any other forms of surgery, and systemic therapies are recommended for these patients [19]. Surgery approaches, such as radiofrequency ablation, liver transplantation, and resection are only effective for nonmetastatic patients with tumor node less than 3 cm, and the recurrence reached 70%, which entails multiple therapeutic paradigms [20]. HCC progresses fast and is often refractory to many chemotherapeutic drugs. Sorafenib has been recommended as the standard of care first line therapy in China, with its safety and modest efficacy been validated in Asian-Pacific populations [12, 21]. Among many other failed attempts to achieve better survival, such as erlotinib, everolimus, brivanib, sunitinib, and doxorubicin. Regorafenib was shown to extend the survivals from 7.8 to 10.6 months for patients tolerant with sorafenib, and thus becomes FDA-approved second-line treatment [22, 23]. However, the benefit of regorafenib in HCC is still limited, and long-term exposure to regorafenib or sorafenib could lead to drug tolerance and subsequent progression.

Recently, various cancer therapies have been developed and testing in human and number of studies of Traditional Chinese medicine (TCM) in cancer has increased rapidly. Traditional Chinese herbal medicines demonstrated antagonistic effect against various cancers, such as colorectal cancer, gastric cancer, and HCC [24–27]. The most sought-after extract of TCM is resveratrol derived from mulberries, peanuts, and grapes, which exhibit inhibitory effect on cancer stem cells of HCC [28]. Gao et al. revealed that resveratrol suppresses human HCC via HGF-c-Met signaling pathway [29]. Marquardt et al. identified that curcumin, an extract from ginger, impaired the oncogenic NF-*κ*B signaling and suppress stemness of liver cancer [30]. Chung et al. showed that curcumin and epigallocatechin gallate could restrain STAT3-NF*κ*B signaling pathway thereby hampering the development of cancer stem cell phenotypes [31]. However, the combined therapy integrating TCM and target therapeutic drugs in HCC population is still lacking.

This study evaluates the effect of DSS-spleen tonics in mid/late-stage HCC patients treated with regorafenib. In the 120 recruited patients, we did not observe significant alteration in safety profile in the group coadministered with DSS-spleen tonics, yet it slightly reduced the incidence of palmar-plantar erythrodysesthesia, the major AE of regorafenib. Regarding the efficacy of DSS-spleen tonics, the TTP was extended slightly but significantly in patients coadministered with regorafenib and DSS-spleen tonics. Compared with patients treated with regorafenib, the median overall survival in DSS group is also longer than REG group. We further validated the antitumor effect of DSS-spleen tonics in HCC cell line HCCLM3 cells and HCCLM3 xenograft mouse model as well. We observed the cell proliferation and invasion were both inhibited by DSS-spleen tonics, and the tumor volume and weight of the mouse model treated with DSS-spleen tonics were decreased. Together, these results demonstrated that DSS-spleen tonics could exert moderate suppressive effect on HCC.

Hypoxia-inducible factor-1*α* was reported to transactivate the VEGF and matrix metalloproteinase-2 (MMP-2), both of which are usually upregulated in a variety of cancers and are key regulator in angiogenesis [32]. The expression of VEGF is highly correlated with Hypoxia-Inducible Factor-1 *α* (HIF-1*α*), MMP-2 and microvessel density (MVD) [33].

At molecular level, we discovered that VEGF, HIF-1*α*, VEGF-2, and MVD were both downregulated by DSS-spleen tonics and regorafenib in HCCLM3 cell line, and cotreatment of both could enhance the effect of single treatment. These results suggest that DSS-spleen tonics function synergistically with regorafenib in HCC by enhancing the regulation of regorafenib on VEGF, MMP-2, HIF-1*α,* and MVD, and may diminish angiogenesis during HCC progression. In the future, we will pay more attention to exploring the mechanism of inhibiting tumor growth [34, 35].

## Figures and Tables

**Figure 1:** Cell viability and Transwell assay of HCCLM3 cells treated with regorafenib and/or DSS-splenic tonics. (a) MTT assay result, absorbance at 570 nm at 24 h, 48 h and 72 h posttreatment; (b) Transwell invasion assay were subjected to detect the migration and invasion capacity of HCCLM3 cells treated with regorafenib and/or DSS.

**Figure 2:** Synergistic effect of combining regorafenib and DSS-splenic tonics. (a). Weight change of HCCLM3 xenograft nude mice model treated with regorafenib (a), DSS-splenic tonics (b), Regorafenib + DSS-splenic tonics (c) and control; (b). Changes of subcutaneous tumor of HCCLM3 xenograft nude mice model treated with regorafenib and/or DSS-splenic tonics; (c). Size of primary tumor of HCCLM3 xenograft nude mice model treated with regorafenib and/or DSS-splenic tonics; (d) Lung metastasis of HCCLM3 xenograft nude mice model treated with regorafenib (REG), DSS-splenic tonics (DSS), Regorafenib + DSS-splenic tonics (REG-DSS) and control. DSS-spleen tonics downregulates VEGF, HIF-1*α*, VEGF-2 and MVD.

**Figure 3:** Immunohistochemistry staining (a), western blot (b) and mRNA quantification (c) of tumors obtained from xenograft mice model treated with regorafenib, DSS-splenic tonics, Regorafenib + DSS-splenic tonics and control.

**Table 1:** Baseline characteristics of patients with hepatocellular carcinoma (*n* = 120).

Characteristics	# of patients
Gender	
Female	28
Male	92
Age, median, years (range)	48 (28–70)
HBV-positive	84 (70%)
HCV-positive	12 (10%)
Alcohol abuse	18 (15%)
ECOG-PS, ≤1	120 (100%)
Child-pugh score	
5	56 (46.7%)
6	42 (35%)
7	15 (12.5%)
Vascular invasion	74 (62%)
Extrahepatic metastasis	36 (30%)
BCLC stage	
B	18 (15%)
C	102 (85%)
AFP	
<400 ng/mL	93 (77.5)
≥400 ng/mL	27 (22.5%)

Safety of regorafenib and combined therapy with DSS.

**Table 2:** Adverse events.

	REG	REG-DSS	*p*-value
Diarrhea	28	30	0.9983
Fatigue	30	33	
Palmar-plantar erythrodysesthesia	40	32	
Elevated serum aspartate aminotransferase	28	27	
Elevated serum blood bilirubin	8	9	
Elevated serum amylase	9	10	
Hypoalbuminemia	18	16	
Hypertension	25	28	
Erythema multiforme	19	21	
Anemia	16	17	
Decreased platelet count	10	11	

Combined therapy of Regorafenib with DSS-spleen tonics achieved better efficacy in mid-/late-stage HCC.

**Table 3:** PFS, TTP, and OS of REG and REG-DSS group patients.

Group	TTP (95% CI)	PFS (95% CI)	OS (95% CI)
REG	6.8 (3.5–9.7)	6.8 (3.5–9.7)	17.2 (11.5–22.8)
Treatment ≥4.2 m	7.1 (5.8–8.6)	7.1 (5.8–8.6)	
Treatment ＜4.2 m	3.7 (2.5–4.8)	3.7 (2.5–4.8)	

REG-DSS	7.3 (4.2–9.9)	7.3 (4.2–9.9)	18.2 (12.6–23.4)
Treatment ≥4.2 m	7.9 (6.8–8.9)	7.9 (6.8–8.9)	
Treatment ＜4.2 m	4.6 (3.2–6.2)	4.6 (3.2–6.2)	

Overall	7.1 (3.9–9.8)	7.1 (3.9–9.8)	17.6 (11.5–22.8)
Treatment ≥4.2 m	7.6 (6.6–8.5)	7.6 (6.6–8.5)	
Treatment ＜4.2 m	4.3 (2.0–6.5)	4.3 (2.0–6.5)	

DSS-spleen tonics had synergistic antitumor efficacy with Regorafenib in HCCLM3 cell line.

**Table 4:** Weight changes of 40 HCCLM3 xenograft nude mice model.

Group		Litter									
		1	2	3	4	5	6	7	8	9	10
*DSS*	Week 0	18	17	18	17	18	17	19	19	17	18
	Week 4	22.5	21.2	22	20.5	22.2	21.8	23.5	23.1	20	22.6

*REG*	Week 0	17	17	18	17	19	18	19	19	17	18
	Week 4	20.6	21	21.7	20.5	22.8	21.5	23	22.9	20.5	21.8

*REG-DSS*	Week 0	17	17	17	17	18	18	18	19	18	19
	Week 4	24.5	25	25.2	24.6	25.9	25.8	25.6	27	26.2	26.9

*Blank*	Week 0	18	18	18	17	19	17	19	19	18	18
	Week 4	21	20.2	20.5	19.2	22	19	21.5	22	20	20.8

**Table 5:** Mean weight at Week 4.

Group	Mean	SD	95% CI
DSS	22.06	0.11	21.84–22.83
REG	21.63	0.11	21.41–21.85
REG-DSS	25.79	0.11	25.57–26.01
Blank	20.38	0.11	20.16–20.61

## Data Availability

The experimental data used to support the findings of this study are available from the corresponding author upon request.

## References

[1] Li T., Xie J., Shen C.. (2016). Upregulation of long noncoding RNA ZEB1-AS1 promotes tumor metastasis and predicts poor prognosis in hepatocellular carcinoma. *Oncogene*.

[2] Ogasawara S., Ooka Y., Itokawa N. (2020). Sequential therapy with sorafenib and regorafenib for advanced hepatocellular carcinoma: a multicenter retrospective study in Japan. *Investigational New Drugs*.

[3] Yang T., Lu J. h., Wu M. c. (2010). Hepatocellular carcinoma in China. *BMJ*.

[4] Nahon P., Vibert E., Nault J. C., Ganne‐Carrié N., Ziol M., Seror O. (2020). Optimizing curative management of hepatocellular carcinoma. *Liver International*.

[5] Sur B. W., Sharma A. (2018). Transarterial chemoembolization for hepatocellular carcinoma. *Journal of Radiology Nursing*.

[6] Zheng L., Guo C.-Y., Chen C.-S. (2017). Sorafenib improves lipiodol deposition in transarterial chemoembolization of Chinese patients with hepatocellular carcinoma: a long-term, retrospective study. *Oncotarget*.

[7] Hinshaw J. L., Lee F. T. (2007). Cryoablation for liver cancer. *Techniques in Vascular and Interventional Radiology*.

[8] Nishikawa H., Kimura T., Kita R., Osaki Y. (2013). Radiofrequency ablation for hepatocellular carcinoma. *International Journal of Hyperthermia*.

[9] Le Grazie M., Biagini M. R., Tarocchi M., Polvani S., Galli A. (2017). Chemotherapy for hepatocellular carcinoma: the present and the future. *World Journal of Hepatology*.

[10] Chen S., Cao Q., Wen W., Wang H. (2019). Targeted therapy for hepatocellular carcinoma: challenges and opportunities. *Cancer Letters*.

[11] Kudo M., Finn R. S., Qin S. (2018). Lenvatinib versus sorafenib in first-line treatment of patients with unresectable hepatocellular carcinoma: a randomised phase 3 non-inferiority trial. *The Lancet*.

[12] Omata M., Cheng A.-L., Kokudo N. (2017). Asia-Pacific clinical practice guidelines on the management of hepatocellular carcinoma: a 2017 update. *Hepatology International*.

[13] Liao Y.-H., Li C.-I., Lin C.-C., Lin J.-G., Chiang J.-H., Li T.-C. (2017). Traditional Chinese medicine as adjunctive therapy improves the long-term survival of lung cancer patients. *Journal of Cancer Research and Clinical Oncology*.

[14] Keji C., Hao X. (2003). The integration of traditional Chinese medicine and Western medicine. *European Review*.

[15] Chi C. (1994). Integrating traditional medicine into modern health care systems: examining the role of Chinese medicine in Taiwan. *Social Science & Medicine*.

[16] Wu X.-N. (1998). Current concept of Spleen-Stomach theory and Spleen deficiency syndrome in TCM. *World Journal of Gastroenterology*.

[17] World Health Organization (2018). *Updated WHO Projections of Mortality and Causes Of Death 2016-2060*.

[18] Younossi Z., Stepanova M., Ong J. P. (2019). Nonalcoholic steatohepatitis is the fastest growing cause of hepatocellular carcinoma in liver transplant candidates. *Clinical Gastroenterology and Hepatology*.

[19] Zucman-Rossi J., Villanueva A., Nault J.-C., Llovet J. M. (2015). Genetic landscape and biomarkers of hepatocellular carcinoma. *Gastroenterology*.

[20] Ishizawa T., Hasegawa K., Aoki T. (2008). Neither multiple tumors nor portal hypertension are surgical contraindications for hepatocellular carcinoma. *Gastroenterology*.

[21] Cheng A.-L., Kang Y.-K., Chen Z. (2009). Efficacy and safety of sorafenib in patients in the Asia-Pacific region with advanced hepatocellular carcinoma: a phase III randomised, double-blind, placebo-controlled trial. *The Lancet Oncology*.

[22] Johnson P. J., Qin S., Park J.-W. (2013). Brivanib versus sorafenib as first-line therapy in patients with unresectable, advanced hepatocellular carcinoma: results from the randomized phase III BRISK-FL study. *Journal of Clinical Oncology*.

[23] Cheng A.-L., Kang Y.-K., Lin D.-Y. (2013). Sunitinib versus sorafenib in advanced hepatocellular cancer: results of a randomized phase III trial. *Journal of Clinical Oncology*.

[24] Abou-Alfa G. K., Niedzwieski D., Knox J. J. (2016). Phase III randomized study of sorafenib plus doxorubicin versus sorafenib in patients with advanced hepatocellular carcinoma (HCC): CALGB 80802 (Alliance). *Journal of Clinical Oncology*.

[25] Bruix J., Qin S., Merle P. (2017). Regorafenib for patients with hepatocellular carcinoma who progressed on sorafenib treatment (RESORCE): a randomised, double-blind, placebo-controlled, phase 3 trial. *The Lancet*.

[26] Wang X., Wang N., Cheung F., Lao L., Li C., Feng Y. (2015). Chinese medicines for prevention and treatment of human hepatocellular carcinoma: current progress on pharmacological actions and mechanisms. *Journal of Integrative Medicine*.

[27] Sun Y.. J.. z.. b.. h., Li T.. l., Liu Z., Zhang G. m., Yao J. c., Li J. (2018). Arctigenin inhibits liver cancer tumorigenesis by inhibiting gankyrin expression via C/EBP*α* and PPAR*α*. *Frontiers in Pharmacology*.

[28] Wang Y., Feng L., Piao B., Zhang P. (2017). Review on research about traditional Chinese medicine in cancer stem cell. *Evidence-based Complementary and Alternative Medicine*.

[29] Efferth T. (2012). Stem cells, cancer stem-like cells, and natural products. *Planta Medica*.

[30] Shankar S., Singh G., Srivastava R. K. (2007). Chemoprevention by resveratrol: molecular mechanisms and therapeutic potential. *Frontiers in Bioscience*.

[31] Gao F., Deng G., Liu W., Zhou K., Li M. (2017). Resveratrol suppresses human hepatocellular carcinoma via targeting HGF-c-Met signaling pathway. *Oncology Reports*.

[32] Marquardt J. U., Gomez-Quiroz L., Arreguin Camacho L. O. (2015). Curcumin effectively inhibits oncogenic NF-*κ*B signaling and restrains stemness features in liver cancer. *Journal of Hepatology*.

[33] Chung S. S., Vadgama J. V. (2015). Curcumin and epigallocatechin gallate inhibit the cancer stem cell phenotype via down-regulation of STAT3-NF*κ*B signaling. *Anticancer Research*.

[34] Wan R., Mo Y., Chien S. (2011). The role of hypoxia inducible factor-1*α* in the increased MMP-2 and MMP-9 production by human monocytes exposed to nickel nanoparticles. *Nanotoxicology*.

[35] Saponaro C., Malfettone A., Ranieri G. (2013). VEGF, HIF-1*α* expression and MVD as an angiogenic network in familial breast cancer. *PLoS One*.

